The article "A land data assimilation system for sub-Saharan Africa food and water security applications" was published in 2017. Journal: Sci Data.

# A land data assimilation system for sub-Saharan Africa food and water security applications

**DOI:** 10.1038/sdata.2017.12

**Published:** 2017-02-14

**Authors:** Amy McNally, Kristi Arsenault, Sujay Kumar, Shraddhanand Shukla, Pete Peterson, Shugong Wang, Chris Funk, Christa D. Peters-Lidard, James P. Verdin

**Affiliations:** 1 University of Maryland Earth Systems Science Interdisciplinary Center, College Park, Maryland 20740, USA; 2 NASA Goddard Space Flight Center, Greenbelt, Maryland 20771, USA; 3 SAIC, Inc., McLean, Virginia 22102, USA; 4 University of California Santa Barbara, Department of Geography and Climate Hazards Group, Santa Barbara, California 93106, USA; 5 U.S. Geological Survey (USGS) Earth Resources Observation and Science (EROS) Center, Sioux Falls, South Dakota 57105, USA

**Keywords:** Hydrology, Natural hazards

## Abstract

Seasonal agricultural drought monitoring systems, which rely on satellite remote sensing and land surface models (LSMs), are important for disaster risk reduction and famine early warning. These systems require the best available weather inputs, as well as a long-term historical record to contextualize current observations. This article introduces the Famine Early Warning Systems Network (FEWS NET) Land Data Assimilation System (FLDAS), a custom instance of the NASA Land Information System (LIS) framework. The FLDAS is routinely used to produce multi-model and multi-forcing estimates of hydro-climate states and fluxes over semi-arid, food insecure regions of Africa. These modeled data and derived products, like soil moisture percentiles and water availability, were designed and are currently used to complement FEWS NET’s operational remotely sensed rainfall, evapotranspiration, and vegetation observations. The 30+ years of monthly outputs from the FLDAS simulations are publicly available from the NASA Goddard Earth Science Data and Information Services Center (GES DISC) and recommended for use in hydroclimate studies, early warning applications, and by agro-meteorological scientists in Eastern, Southern, and Western Africa.

## Background & Summary

Using rainfall and other meteorological inputs (temperature, humidity, radiation, and wind), the Famine Early Warning Systems Network (FEWS NET) Land Data Assimilation System (FLDAS) produces multi-model and multi-forcing estimates of hydro-climate conditions such as soil moisture, evapotranspiration, and runoff. The FLDAS system was created under a NASA Applied Sciences Program Water Resources grant as a collaboration between the U.S. Geological Survey (USGS) Earth Resources Observation and Science (EROS) Center, NASA Goddard Space Flight Center (GSFC), and the University of California Santa Barbara (UCSB) Climate Hazards Group (CHG). The FLDAS variables are relevant to agricultural and water resource monitoring and are used to produce indices, like soil moisture percentiles, that show how current hydrologic extremes compare to conditions observed over the past 30+ years. Within FEWS NET, FLDAS outputs are combined with remotely sensed estimates, ground observations, and reports from the field to identify potential food security crises. FEWS NET reports^1,2^ regarding the 2015 Ethiopia Drought and 2015–16 Southern Africa drought are examples of this approach. Using multiple sources of information typifies the FEWS NET ‘convergence of evidence’ framework^3^ for characterizing agricultural conditions and providing early warning for food emergencies.

The ideal gridded land surface model (LSM) dataset for food and water security monitoring would be (1) driven by a rainfall product that performs well over data sparse food insecure regions; (2) available over a long historical record and near-real time for contextualizing current events and initializing forecasts; and (3) useful for both the drought monitoring and hydrological science communities by providing estimates of land surface states and fluxes that can be used to further our understanding of drought dynamics and impacts. At present, the Global Land Data Assimilation System (GLDAS)^4^ does provide a suite of outputs at 1-month latency over a global domain, but relies on global rainfall products (specifically CMAP^5^ and Princeton^6^) that have not been optimized for data sparse, food insecure regions. From the drought monitoring community there are existing efforts like Africa Flood and Drought Monitor (ADFM)^7^. There are also global efforts: the Global Integrated Drought Monitoring and Prediction System (GIDMaPS)^8^, the UN Food and Agriculture Organization (FAO) Global Information and Early Warning System on Food and Agriculture (GIEWS), and the Global Drought Information System Portal^9^. To complement these efforts and better meet the needs of food and water security monitoring, the FLDAS provides (1) flexible use of different forcing products, including FEWS NET operational rainfall, (2) multiple land models, (3) routine evaluation, and (4) rapid and convenient data distribution. By relying on standard FEWS NET rainfall inputs FLDAS maintains consistency between the different FEWS NET drought metrics. This allows FEWS NET and FEWS NET partners to better harness the expertise of agro-climate scientists and food security analysts. This spatially distributed (African, American, and European) team of experts can provide feedback on the relationship between field observed crop conditions, remotely sensed, and modeled hydro-meteorological variables.

FLDAS’s capacity to use different land models, rainfall, and meteorological inputs allows FEWS NET to bracket model- and forcing-related uncertainty. FLDAS’ provision of physically meaningful quantitative information (e.g., runoff) can also be used to better characterize hydrologic drought and water availability. This is important given that water insecurity may often exacerbate food insecurity. Finally, this dataset (as highlighted in the Usage Notes section) can be used in conjunction with remotely sensed estimates e.g., evapotranspiration, to make effective characterizations of agricultural drought conditions and provide routine drought evaluations. An additional feature of the FLDAS is that these data can be visualized using the Giovanni online tool^10^ (http://giovanni.gsfc.nasa.gov/giovanni/) or downloaded from the NASA Godard Earth Sciences Data and Information Service Center (GES DISC), allowing researchers to ask questions and explore FLDAS outputs. Subsets of this data can also be easily compared with other indicators using the Early Warning eXplorer (http://ewx.chg.ucsb.edu:8080/EWX/index.html), and downloaded from the USGS FEWS NET Data Portal (http://earlywarning.usgs.gov/fews).

Figure 1 shows the NASA Land Information System (LIS) framework’s^11,12^ customized instance of FLDAS with three main components: (1) meteorological and parameter inputs, (2) LSMs, and (3) post-processing for evaluation, calculation of drought indices, and archiving over three domains in Africa. Table 1 provides more specifics about the FLDAS specifications. In this Data Descriptor’s Methods section, we explain in detail the FLDAS LSMs and their parameters, meteorological inputs, FLDAS model configuration and outputs, and LIS software code availability. The Data Records section provides details about the FLDAS monthly archive and repository. The Technical Validation section includes FLDAS comparisons with reference rainfall, soil moisture, and evapotranspiration datasets. We conclude with Usage Notes, which describes the FLDAS data and the interactive NASA Giovanni data interface, applied in different ways to assess the 2015–16 Southern Africa drought.

## Methods

Most livelihood systems monitored by FEWS NET are based on subsistence agriculture and pastoralism, and consequently are vulnerable to hydroclimatic extremes, especially drought. For this reason, weekly assessments of growing season conditions are made using the latest monitoring and weather forecast products from NASA, USGS, UCSB CHG and the National Oceanic and Atmospheric Administration (NOAA). Remote sensing estimates of precipitation, vegetation, and snow are operationally ingested by USGS and UCSB CHG from NASA and NOAA and used to make a variety of information products, including mapped estimates of anomalous precipitation, vegetation, crop water satisfaction, soil moisture, snow cover, snow water equivalent, runoff, and stream flow. The FLDAS was created to help streamline and add consistency to this process. It includes the domains, data streams, and monitoring requirements associated with food security assessment in data-sparse, developing countries in Africa. The goal is to make more effective use of limited available hydroclimatic observations through the LIS framework’s data management and modelling capabilities.

### NASA LIS

The NASA LIS framework is designed for high performance terrestrial hydrologic modelling, with development led by the Hydrological Sciences Laboratory at NASA Goddard Space Flight Center (GSFC). LIS is structured to enable community sharing, the reuse of modelling tools and data resources, and promote transitioning the latest Earth science research into operations. Specifically, the LIS framework includes the Land Data Toolkit preprocessor, the Land Information System core modules, and Land Verification Toolkit post processor. The LIS framework is the software that underpins the FLDAS, and, similarly, is used in other successful products like the NASA Global Land Data Assimilation System (GLDAS)^4^ and the North American Land Data Assimilation System (NLDAS)^13^. As an instance of the LIS, FLDAS uses specific features from each of these components, which we will explain in more detail.

The LSMs in FLDAS require a large suite of time-invariant and climatological land surface parameters such as vegetation, soils and topography, among others (Table 2). The Land Data Toolkit (LDT; http://lis.gsfc.nasa.gov/documentation/ldt) is a data pre-processing environment for different LSMs that enables specification of these parameters (Fig. 1).

Routine evaluation of the FLDAS outputs is conducted using the Land Verification Toolkit (LVT)^14^ (Fig. 1), which supports both direct comparisons of the model outputs against independent (ground/satellite) measurements and indirect comparisons such as lagged ranked correlation of soil moisture against vegetation indices^15^. In addition, LVT also computes metrics of hydrologic extremes such as soil moisture percentiles, by quantifying the departures of the model estimates relative to the long-term model climatology.

### FLDAS land surface models and parameters

#### VIC

The Variable Infiltration Capacity (VIC)^16^ spatially distributed macroscale hydrology model has been widely used at global and regional scales and has been demonstrated to accurately capture the hydrology of different regimes^17–19^. The inclusion of VIC version 4.1.2 (VIC4.1.2) in the FLDAS was intended to promote interactions between research and applications. It is the main water balance model used by the Princeton Africa Flood and Drought Monitor^7^ and has been introduced to FEWS NET for seasonal hydrologic forecasting applications^20^. In contrast to these applications, however, FLDAS uses VIC4.1.2 in energy and water balance mode. The purpose of this is to better represent surface fluxes in environments where evapotranspiration (ET) is a greater proportion of rainfall than runoff. The water balance simulation mode, run at a daily time step, does not solve the energy balance, eliminates the ground heat flux solution, and assumes that the surface temperature is equal to the air temperature. In contrast, the energy and water balance simulation mode, run at a sub-daily time step, closes the energy balance though an iterative process that adjusts surface temperature and surface energy fluxes (sensible heat, latent heat, ground heat, outgoing long wave radiation) to balance incoming radiation. There is a comparison of VIC simulation modes for the Rhine River^21^ and additional explanation and comparisons can be found as a technical note on the University of Washington VIC website http://www.hydro.washington.edu/Lettenmaier/Models/VIC/Documentation/TechnicalNotes/Modes.shtml.

Evapotranspiration in VIC4.1.2 (and Noah3.3) includes three components: canopy-intercepted evaporation, transpiration from vegetation canopies, and evaporation from bare soil. Total evapotranspiration is the sum of these components, weighted by respective land surface coverage fractions.

In VIC4.1.2, reference ET (RefET) is calculated using the Penman-Monteith equation. Canopy transpiration is calculated by scaling RefET with canopy resistance. Canopy-intercepted evaporation is calculated by scaling RefET with the canopy architectural resistance for humidity and the aerodynamic resistance for heat and water. The bare soil, or direct, evaporation is calculated by scaling RefET by current soil moisture conditions, wilting point soil moisture, and field capacity.

In VIC4.1.2, the surface runoff is determined by subtracting the precipitation and the infiltration capacity of the top (0–10 cm) soil layer. The subsurface runoff is computed as a nonlinear stepwise function of excess soil moisture from the bottom soil layer, as firstly introduced in the Arno model formulation^22^.

VIC4.1.2 parameter inputs (Table 2) include soil textures and bulk density^23^, and soil characteristic curve parameters^24^, monthly climatology leaf area index^25^, the University of Maryland landcover classification^26^ from the Advanced Very High Resolution Radiometer (AVHRR), and other vegetation parameters^7,18,27^.

#### Noah

The Noah Land Surface Model^28^ is a four soil-layer water and energy balance LSM. It is a widely used model by both operational and research communities. For example, Noah is the operational LSM in the NOAA National Centers for Environmental Prediction (NCEP) weather, climate and data assimilation systems and at the US Air Force 557th Weather Wing. There are a number of examples of Noah being used over different domains in Africa, e.g., West Africa^29,30^, Volta Basin^31^, East Africa^32,33^ and coupled with the Weather Research and Forecasting (WRF) model for West Africa^34^ and Kenya^35^. The FLDAS uses the Noah LSM version 3.3 (ref. 36). Later versions of Noah have been implemented in LIS and may be used in the future if the model physics, or other features are determined to improve water and energy balance estimates for FEWS NET domains of interest.

Like VIC4.1.2, Noah3.3’s total evapotranspiration is the sum of canopy intercepted water evaporation, transpiration from vegetation canopies, and evaporation from bare soil, weighted by respective land surface coverage fractions. Different from VIC4.1.2, Noah3.3’s potential evapotranspiration (PET) is calculated using the Penman approach, which assumes saturated ground surface and no canopy resistance. Transpiration is calculated by scaling PET with solar radiation, vapor pressure deficit, air temperature and soil moisture. Evaporation of canopy-intercepted water is calculated by scaling PET by intercepted canopy water content and the maximum canopy capacity. The bare soil evaporation is calculated by scaling PET by a factor of current soil moisture availability.

In Noah3.3, Surface runoff is computed using a two-layer conceptual approach developed by Schaake *et al.*^37^ from the Simple Water Balance (SWB) model. The upper layer is a shallow bucket that produces surface runoff from excess precipitation when there is no soil moisture deficit. Subsurface runoff is produced as gravitational drainage from the bottom soil layer, which is calculated using Darcy’s equation.

FLDAS-Noah3.3 parameter inputs (Table 2), include the NCEP modified International Global Biosphere Project (IGBP)^38,39^ landcover map from the MODerate resolution Imaging Spectrometer (MODIS) landcover classification, monthly minimum and maximum greenness fraction^40^, and albedo maps^41^. These data, as well as hybrid STATSGO/FAO soil texture data sets, and vegetation and soil parameters tables are maintained by the Research Application Laboratory (RAL) and are available at http://www.rap.ucar.edu/research/land/technology/lsm.php.

### Meteorological inputs

FLDAS models use FEWS NET specific rainfall products, but also require additional meteorological inputs (e.g., temperature, humidity, radiation, and wind). To generate low-latency products FLDAS uses NOAA Global Data Assimilation System (GDAS)^42^ 3-hourly meteorological inputs available from 2001-present at<1-day latency. For a longer historical record FLDAS uses NASA’s Modern Era Reanalysis for Research and Applications version 2 (MERRA-2)^43^ (1979-present) 1-hourly products with a two-week latency.

Rainfall, as mentioned earlier, and described in detail later, is the most important input to the FLDAS. Temperature is also particularly important for both the water and energy balance. MERRA-2 provides a long record, sub-daily time step and has been shown to agree well, in terms of daily and annual bias (0–1 K) with CRU^44^ temperature estimates^43^. We compared monthly MERRA-2, GDAS and GLDAS temperature estimates (2001–2010, not shown) over our Southern, Eastern and Western Africa domains and found that all three products are well correlated (r>0.7). However, GDAS has a noticeable low bias (about 1 K) until ~2007 compared to MERRA-2 and GLDAS temperature fields. From 2007-present, MERRA-2 and GDAS temperatures continue to be well correlated and have a similar mean.

#### RFE2

The African Rainfall Estimation version 2.0 (refs 5,45) (RFE2) rainfall product is from the NOAA Climate Prediction Center (CPC). RFE2 is derived from satellite (infrared and microwave) observations and blended with World Meteorological Organization Global Telecommunication Stations (GTS) data. It is available from 2000 to present at 0.1° latitude/longitude (approximately 10 km^2^) at a 1-day latency (Table 3). Examples of RFE2 evaluation have been conducted for Burkina Faso^46^, Western Africa^47–49^, Mozambique^50^, the Nile Basin^51^, and Eastern and Southern Africa^52,53^. In addition to research applications, FEWS NET analysts use RFE2 operationally to track weather hazards on a weekly basis. More information is available at the CPC International Desk website under ‘Africa’ (http://www.cpc.ncep.noaa.gov/products/international/africa/africa.shtml).

#### CHIRPS

The Climate Hazards group Infrared Precipitation with Stations (CHIRPS)^54^ dataset is an IR-station blended rainfall product that has been bias-corrected with monthly station climatologies, i.e., CHPclim^55^. CHIRPS is available at the daily, pentadal (~5-day), dekadal (~10-day), and monthly time step, quasi-global (60S-60N), 0.05 degrees spatial resolution (Table 3) designed for drought monitoring. CHIRPS is released about 2-weeks after then end of the previous month (i.e., August 1–31 daily CHIRPS is available on September 15th). CHIRPS has been evaluated for Burkina Faso^46^, Mozambique^50^, the Nile Basin^51^, and continental Africa^54^. On-going evaluations can be found at the UCSB Climate Hazards Group website (http://chg.ucsb.edu).

### Sub-daily disaggregation of rainfall

For agricultural drought monitoring applications daily, dekadal, and monthly rainfall totals are favoured by decision makers^56^. In contrast, the LSMs that solve both the energy and water balance are run at hourly or finer time steps (e.g., Noah3.3 at 30-minutes and VIC4.1.2 at 1-hour), requiring sub-daily rainfall inputs. To meet the needs of these LSMs, we developed a new module using the Land Data Toolkit (LDT) pre-processor to temporally disaggregate the daily RFE2 and CHIRPS rainfall, using an approach similar to the North American LDAS (NLDAS) precipitation downscaling method^57^. For this approach, we assume that the finer timescale, reference dataset, e.g., 3-hourly GDAS precipitation, represents an accurate diurnal cycle. First we derive sub-daily (e.g., 3-hourly) disaggregation weights that represent the proportion of the 24-hour total precipitation that fell during the sub-daily period. If the total is zero in a area of non-zero precipitation then uniform weighting spreads precipitation evenly throughout the day. The daily rainfall is then multiplied by the weights to arrive at the temporally disaggregated fields. Since the reference dataset is only used to derive the disaggregation weights the daily summation preserves the total from the daily rainfall product. This new sub-daily time series is then used as the final FLDAS precipitation input. Future work, particularly that involves higher spatial and temporal applications of FLDAS outputs, should explore the accuracy of the sub-daily rainfall distribution of a reference dataset.

### FLDAS model configuration and outputs

Meteorological inputs provided in their native resolution often do not match the spatial and temporal resolution of other datasets, or the resolution at which the user wishes to run the model. One of the important features of the LIS framework is its ability to match spatial and temporal grids at runtime. We have specified the LIS model spatial resolution to match the 0.1°×0.1° RFE2 and CHIRPS rainfall inputs. However, the MERRA-2 has horizontal resolution of 0.5° latitude×0.625° longitude, and the GDAS grid varies over time and is currently at approximately 0.2° (Table 3). We have chosen a bilinear interpolation option in LIS to spatially downscale non-precipitation fields. Using the method developed by the NLDAS^57^, the Noah-GDAS experiments have an environmental lapse-rate correction applied to surface pressure, humidity and downward longwave radiation. At the time of writing, VIC4.1.2 and MERRA-2 experiments did not have this capability. While this introduces some error, the implications for the 0.1 degree Africa domain are relatively minor compared to regions with steep topography and finer spatial resolution. Future versions of the VIC-GDAS and Noah-MERRA-2 experiments will include the topographic adjustment. All of the sub-daily inputs are linearly interpolated to 30-minute and 1-hour model timesteps for Noah3.3 and VIC4.1.2, respectively. Table 4 lists the routine FLDAS outputs and their units. At the time of writing, both FLDAS_A (RFE2+GDAS; Data Citation 1–6) and FLDAS_C (CHIRPS+MERRA-2; Data Citation 7–11 and Data Citation 12) outputs are updated on the NASA GES DISC once a month (see Data Records).

### Soil moisture percentiles

Soil moisture percentiles are indicators of deficits or excesses of land moisture states relative to historical distributions. The percentiles are calculated using the Land Verification Toolkit (LVT)^14^ using soil moisture outputs from Noah3.3 and VIC4.1.2 simulations. First, the soil moisture climatology is generated, using daily gridded outputs from model simulations. The climatology for a particular calendar day is the list of rainfall estimates over all years (start year to 2015) in a 5-day moving window (2 previous days, current day, and 2 next days. For example, the Jan 3 climatology groups Jan 1 to Jan 5 for each year 1982, 1983, 1984,... to 2015 (5 days×33 years=165). Next, the percentile of each day's rainfall estimate is computed using that day's climatology. Finally, the computed daily values are averaged to produce monthly percentile estimates.

### Code availability

The LIS framework software is available as open source under the NASA Open Source Agreement (NOSA) and available at http://lis.gsfc.nasa.gov. This software has been compiled and run on Linux PC (Intel/AMD based) systems and Cray systems. Specific Fortran and C compilers are required, as are several other software libraries, e.g., the Earth System Modeling Framework^58^ and NetCDF. More details are available from the LIS Users Guide, available on the LIS website (https://lis.gsfc.nasa.gov/documentation/lis).

## Data Records

Monthly FLDAS outputs are available from the NASA Goddard Earth Science Data and Information Service Center (GES DISC; http://disc.sci.gsfc.nasa.gov/uui/datasets?keywords=FLDAS) in NetCDF format. There are six experiments available for each domain and land model, with the rainfall and other meteorological inputs listed below:

FLDAS_A_[NOAH01, VIC025]=RFE2+GDAS (2001-present) (Data Citation 1–6).

FLDAS_C_[NOAH01, VIC025]=CHIRPS+MERRA2 (1982-present) (Data Citation 7–12).

At the time of writing, both FLDAS_A and FLDAS_C monthly products are updated at the beginning of the month, e.g., June FLDAS_C and July FLDAS_A data are available at the beginning of August. The FLDAS_C is the recommended product for research applications. On-going work will make FLDAS products available at the same latency as CHIRPS and RFE2 rainfall inputs.

The FLDAS monthly data can also be accessed via the following methods:

- HTTP: Direct download of FLDAS data over the Web. http://hydro1.sci.gsfc.nasa.gov/data/s4pa/FLDAS/
- Mirador: Search and download FLDAS data using the GES DISC search tool. https://mirador.gsfc.nasa.gov/
- OPeNDAP: Download parameter- and spatially-subset data in NetCDF, binary or ASCII text. http://hydro1.sci.gsfc.nasa.gov/opendap/hyrax/FLDAS/
- Giovanni: Online visualization, analysis, and inter-comparison of FLDAS data products. http://giovanni.sci.gsfc.nasa.gov/
- Discover Earth Science Data: Search NASA Earth Science data by keyword and filter by time or space. https://search.earthdata.nasa.gov/
- The USGS FEWS NET data portal: FLDAS Noah+CHIRPS+MERRA-2 (Data Citation 8–10) soil moisture and anomalies are available for Eastern, Southern, and Western Africa. Images can be viewed and downloaded in.png and.pdf formats and data can be downloaded as.tif. http://earlywarning.usgs.gov/fews

## Technical Validation

Development of high quality hydro-meteorological data sets and conducting evaluations of these datasets is inherently challenging over data sparse regions. Product development continues to improve through improved sensors, algorithms and data fusion efforts. For product evaluation FEWS NET relies on a convergence of evidence approach—the use of multiple inputs, and by transforming rainfall inputs into estimates of, for example, soil moisture and evapotranspiration. With that, we are increasing the opportunities for comparison with other products like remotely sensed microwave soil moisture and remotely sensed thermal-ET. Evaluation is an on-going process as new products are developed, and different applications require different metrics—e.g., some products may be better for drought monitoring, while others for flood forecasting.

### Rainfall input evaluation

In addition to the precipitation evaluations mentioned previously (Methods; Meteorological Inputs), we compare here RFE2 and CHIRPS (2001–2010) to a reference dataset: the Global Precipitation Climatology Centre (GPCC) gridded monthly station product^59,60^.

Following the methods in Funk *et al.*^54^, metrics are computed on a per-pixel basis for the rainy-season (defined as the three-wettest months). Using GPCC as the reference dataset, we computed the Pearson correlation coefficient^61^, bias ratio (Bias=Σ Input_rainfall/ΣGPCC) and mean absolute error (MAE=(1/N Σ|(Input_rainfall—GPCC)|)). Figure 2a,b show similar spatial patterns and magnitude for CHIRPS and RFE’s correlation with GPCC. RFE2 has higher correlations in southern and western Africa, while CHIRPS shows higher correlations in Ethiopia. Figure 2c,d show bias ratio, with CHIRPS tending to have a neutral or wet bias compared to GPCC, while RFE2 has a dry bias over eastern Africa and a wet bias over parts of the Sahel. Figure 2e,f show similar patterns in mean absolute error (mm per 3-month accumulation), with CHIRPS having less error in Ethiopia, and parts of Kenya, Tanzania, Mozambique, Zambia, and Niger. While RFE2 has less error in eastern South Africa and Zimbabwe, correlations tend to be lower over the humid forests of central Africa, which is important for broader applications, but this is not a domain included in routine FEWS NET drought monitoring. This lower correlation may be due to CHIRPS being an IR-only (no routine microwave inputs) product, a necessary prerequisite for its long period of record. The fixed cloud detection threshold used in the CHIRPS might be another factor, resulting in poor detection of warm rainfall events in humid areas of the tropics and sub-tropics.

### Soil moisture and evapotranspiration validation results

We compared monthly estimates of FLDAS-simulated soil moisture and evapotranspiration to equivalent remotely sensed observations using pixel-wise anomaly correlation.

For the soil moisture comparison we used the European Space Agency’s Climate Change Initiative soil moisture version 2.2 (CCI-SMv2.2)^62–64^, which is a merged passive and active microwave estimate of near-surface soil moisture (1979–2015). In general, we find that soil moisture estimates derived from CHIRPS (using either Noah3.3 or VIC4.1.2) have higher monthly anomaly correlation with CCI-SMv2.2 than those derived from RFE2 rainfall inputs. The reason for this will require further research, but we hypothesize that the cause is related to the use of country-specific station data for bias correction in CHIRPS while no such station data is used in RFE2. We also found that Noah3.3 soil moisture has higher correlations with CCI-SMv2.2 than that of VIC4.1.2. These results are consistent with previous work over East Africa by McNally *et al.*^65^, and work comparing Noah and VIC in the U.S. (ref. 66). We also stratified correlations by vegetation type, and found particularly low correlations in pixels classified as permanent wetland. This can be attributed to microwave soil moisture retrievals’ ability to detect persistent wetness, while wetlands are not represented in FLDAS models. Figure 3a–c show anomaly correlations between monthly Noah3.3+CHIRPS+MERRA-2 soil moisture (0–10 cm) and CCI-SMv2.2 soil moisture for the years 1992–2015. We used this time period based on analysis performed in East Africa by McNally *et al.*^65^ Considering all months (Jan-Dec) Eastern and Southern Africa are well correlated (r>0.5) while correlation is less (r=0.3–0.5) in Western Africa. We found that the modeled and observed seasonal cycles (start of season, peak, recession) were sometimes out-of-phase, likely because, as other studies have found, the default Noah LSM soil parameterization is not optimal for representing runoff and soil moisture dynamics in West Africa^34^. Data users should note that we found improved correlations when the analysis is conducted on individual months, particularly during the rainy season.

For ET evaluations we used ET anomaly estimates from the Operational Simplified Surface Energy Balance^67^ (SSEBop) model. The SSEBop product provides percent of normal (PON) ET anomalies using a 2003–2013 baseline and is updated once a month, which is important for routine comparisons with FLDAS. Using the same 10-year baseline, we computed the PON for each month with the FLDAS ET products and then performed pixel-wise anomaly correlation. We show anomaly correlations of the Noah3.3+CHIRPS+MERRA-2 estimated ET. There are moderate correlations (r=0.4–0.75) in East Africa (Fig. 4a) and Southern Africa (Fig. 4b), however, in West Africa correlations between these two products were relatively low (r<0.5) (Fig. 4c). Similar correlations were found with VIC ET anomalies. For further investigation we computed 1-month lagged rank correlation of FLDAS ET’s and MODIS NDVI (not shown) and found high correlations (r>0.7) for vegetated pixels. Inspection of the SSEBop time series at sparsely vegetated pixels in Niger and Senegal showed ‘jumpy’ behaviour (e.g., long periods at 100% of normal with spikes to 250%), suggesting that energy balance characteristics of parts of the West Africa domain may result in instability of SSEBop PON algorithm. Similar to the soil moisture comparisons, correlations for individual months tended to be higher during the rainy season (not shown). Additional investigation is needed to further explain the contribution of both the LSM model physics and SSEBop datasets to low correlations in West Africa.

## Usage Notes

In this section we present a sample application of the FLDAS outputs for the 2015–16 drought in Southern Africa. The historic record, low to moderate latency, 10 km resolution, and potential to compute a variety of drought indicators make FLDAS suitable for assessing agricultural and hydrologic drought conditions. We demonstrate how FLDAS can be used to support humanitarian relief efforts and put current water availability conditions in historic context. Southern Africa is known to be vulnerable to El Niño-induced hot and dry conditions^68^. Two consecutive dry years are threatening hydropower and irrigation schemes that have been critical for advancing development in the region^69^. CHIRPS rainfall and FLDAS-derived estimates of water availability anomalies have been used to illustrate the extent and severity of the Southern Africa 2015–16 drought^1^. In this sample application of FLDAS we i) compare how remotely sensed and modeled ET anomalies represent the extent of the drought in February 2016; ii) compare the FEWS NET operational drought index with soil moisture percentiles derived from FLDAS; iii) show how FLDAS experiments represent water availability over short and long time scales; and iv) show how FLDAS outputs can be accessed via GIOVANNI for user-friendly data interaction.

### Context—2015–2016 Southern Africa drought

Southern Africa relies on agriculture for food and income and reservoirs for hydropower production, municipal water supplies, and irrigation. The strong El Niño conditions in 2015 resulted in a late start to the Southern Africa rainy season, high temperatures, and below average rainfall totals. These severe drought conditions across the region negatively impacted crop and pasture growth^1^. While not an El Niño year, the 2014–15 season was characterized by anomalous dryness with low seasonal rainfall totals that negatively impacted crop growth and reservoir storage^70^.

### Comparison with operational ET estimates

First, we compare SSEBop and FLDAS ET anomalies (Data Citation 8) for February 2016 (Fig. 5). The broad spatial patterns from the two products agree in the extent and severity of the dry conditions. Both ET anomaly estimates show strong ET deficits in central South Africa, Swaziland, Lesotho, southern Mozambique, southern Madagascar, south east Zambia, and western Botswana. Both estimates also show normal or above normal ET in Northern Mozambique, Tanzania, and southern Kenya. Given that these ET anomalies are derived from independent estimates, analysts can have confidence in the direction of the anomaly in locations where the products agree, consistent with FEWS NET’s convergence of evidence approach. However, the two estimates do not agree in all locations. Eastern Botswana, for example, is a crop-growing region where SSEBop shows strong deficits while FLDAS ET shows positive anomalies. In this case, analysts would consider additional sources of evidence, like NDVI, rainfall totals, and field reports. For example, the GEOGLAM Early Warning Crop Monitor, which convenes international experts to discuss different data sources, concluded in a February report that sorghum growing conditions were poor in Eastern Botswana^71^. Positive anomalies in FLDAS ET could be attributed to errors in rainfall inputs, or the ET parameterization’s relative lack of sensitivity to temperature inputs. Future work could use both of these datasets to explore the relative roles of temperature and rainfall in drought.

### Rainfall derived agricultural drought indicators

We next show two agricultural drought indictors, derived from rainfall, that provide insight into the overall performance of the 2015/16 growing season. First, 2016 End-of-Season (EOS) Water Requirement Satisfaction Index (WRSI) (Fig. 6a), computed with CHIRPS rainfall and USGS EROS reference ET^72^, where actual ET was consistently less than reference ET, indicating that there was widespread failure or no start of season across Botswana, Namibia, South Africa, and Southern Mozambique. The late or complete lack of start to the rainy season was anticipated to (and did) have severe negative consequences for agricultural outcomes^70^. Figure 6b is a drought classification based on February Noah3.3+CHIRPS+MERRA-2 (Data Citation 8) soil moisture percentiles (0–10 cm). The soil moisture percentiles do indicate widespread negative moisture anomalies with some pockets of extreme drought in eastern South Africa, southern Madagascar, Swaziland, and southern Malawi. February soil moisture percentiles, however, also reflect that Southern Africa monthly rainfall totals were average for January and February. The EOS WRSI metric, on the other hand, is designed to reflect deficits during critical periods, like the crop sowing period in December, which was very dry. These differences in the seasonal representation explain why the EOS WRSI and February soil moisture percentiles show different spatial patterns, despite being driven by the same rainfall inputs.

### Water availability

To characterize water availability during the Southern Africa 2015–16 drought we compute the Standardized Runoff Index (SRI)^73^ with FLDAS runoff. The SRI is calculated by first fitting a gamma distribution to a given historical time series of runoff (the historical time series at each pixel). Probability values are then calculated from the gamma distribution function for each value in the time series. Finally, the SRI for each probability value is computed (using SciPy stats.norm.ppf) as the inverse cumulative distribution function of a standard normal distribution. The SRI values obtained will approximately have zero mean and unit standard deviation. The one-month SRI-1 considers conditions of the current month (April 2016) while the 24-month SRI categorizes conditions for the current and previous 23 months. The map of one-month SRI (Fig. 7a) indicates that runoff is 0.5 to 3 deviations below average across much of the domain. The one-month time scale is relevant to the growing season of a rainfed crop and has a spatial pattern as similar to the evapotranspiration anomalies, drought classification based on soil moisture percentiles, and the WRSI. Water supply reservoirs, on the other hand, are designed to store water between rainy seasons to provide stable supply for different uses such as irrigation, hydropower, and municipal uses like drinking and sanitation. A longer-term index is more appropriate for characterizing how these needs may be impacted by (hydrological) drought. The 24-month SRI (Fig. 7b) shows that water reserves were likely impacted in Lesotho, Swaziland, South Africa, central and northern Mozambique, as well as Malawi and Zimbabwe. This interpretation of the SRI-24 corresponds well with reported^74^ extremely low reservoir levels across the region.

Time series of SRI-24, spatially averaged over the Zambezi basin above the Kariba reservoir (Fig. 8a) (west of 28.76 E) and the Maputo Basin, shared by Swaziland, South Africa and Mozambique (Fig. 8b), further demonstrates that 2015–16 ranks as one of the lowest runoff years in the past 30 years, comparable to severe droughts in 1994–95 and 2004–05. These time series also demonstrate the utility of FLDAS multiple-model and multiple-forcing features. In general the Noah3.3 and VIC4.1.2 runoff generated from the same forcings strongly agree (Fig. 8a,b) suggesting, for relative comparisons of runoff based drought indicators in this region, that model differences contribute negligible uncertainty. However, differences in the forcings, can result in considerable differences in SRI both from contributing data (e.g., CHIRPS has more ground observations and bias correction, RFE2 includes microwave retrievals) as well as the length of the record. For example, the RFE2+GDAS record does not include the 1994–95 drought. Caution should also be used with aggregating over 24-months with the relatively short 2001–2016 record. With respect to forcing data, continued evaluation, e.g., with respect to streamflow observations, can provide information regarding the accuracy of the input datasets.

### Data visualization with NASA’s Giovanni

The NASA GES DISC provides tools for data exploration and visualization through the Giovanni interface (Fig. 9a). This allows users to explore the data before downloading and analysing on their own machines. This example selects rainfall and air temperature from a domain in Southern Africa (Fig. 9b) that was impacted by the 2015–16 drought. We selected a spatial average and time series of December conditions from 1982–2015. Plots can be generated and downloaded as image files (for example, .png, .jpeg, or .pdf) for individual variables, or the data from the plot can be downloaded and imported into a program of the user’s choice. Figure 10 shows a drought index (rainfall—temperature) plotted in rank order to visualize agrometerological conditions during the critical month of December (1982–2015). 2015 had the combined hottest and driest conditions on record, while 2007 had the combined coolest and wettest conditions.

### Summary

The FLDAS dataset presented here has been designed for drought monitoring in Africa where it is essential to (1) compare different modelled and remotely sensed datasets for accurate characterization of droughts, and (2) place current conditions in historical context for humanitarian decision support. While similar to other global land modelling or Africa drought monitoring systems, the FLDAS uses operational (RFE2) and research (CHIRPS) FEWS NET precipitation products to provide both low latency and research quality estimates, respectively. Meanwhile, choice of evaluation methods and derived drought indices are guided by the needs of food and water security analysts. Moreover, being an instance of the NASA LIS framework affords the potential to leverage other hydrological research and software development projects. In particular, soil moisture data assimilation and seasonal forecasting capabilities are being developed for several LIS-based projects that may benefit FLDAS in the future. While improvements to FLDAS are already being made, e.g., improved latency to better track conditions as they are evolving, the current data products are well suited for characterizing the spatial extent and providing historical context to drought conditions.

## Additional Information

**How to cite this article:** McNally, A. *et al.* A land data assimilation system for sub-Saharan Africa food and water security applications. *Sci. Data* 4:170012 doi: 10.1038/sdata.2017.12 (2017).

**Publisher’s note:** Springer Nature remains neutral with regard to jurisdictional claims in published maps and institutional affiliations.

## Supplementary Material



## Figures and Tables

**Figure 1:** Schematic of the Famine Early Warning Systems Network (FEWS NET) Land Data Assimilation System (FLDAS). The Land Data Tool Kit (LDT) is used to pre-process FLDAS landcover parameters from the IGPB and UMD classification derived from the MODIS and AVHRR instruments, respectively. If required to solve energy balance equations, LDT transforms daily RFE2 and CHIRPS rainfall into sub-daily inputs for the land surface models. Additional meteorological inputs are from GDAS and MERRA-2. FLDAS includes Noah3.3, VIC4.1.2 and GeoWRSI models, which are run over three domains in Africa, and produce estimates of hydrologic states like soil moisture (SM) and fluxes like runoff (RO), evapotranspiration (ET) and streamflow. Model outputs are used as inputs to the Land Verification Toolkit (LVT) for evaluation or generation of drought indices. Evaluation includes remotely sensed ET anomalies from the Operational Simplified Surface Energy Balance (SSEBop) model, soil moisture from the European Space Agencies Climate Change Initiative (CCI-SMv2.2) and the Normalized Difference Vegetation Index (NDVI), as well as *in-situ* observations from the Global Runoff Data Center (GRDC). FLDAS routinely computes soil moisture percentiles, and has capabilities to compute the Standardized Precipitation Index (SPI), Standardized Soil Water Index (SSWI) and others. Monthly FLDAS outputs are available via the UC Santa Barbara Early Warning eXplorer (EWX), and different NASA Goddard Earth Science Data and Information Services Center (GES DISC) interfaces.

**Figure 2:** Comparison of CHIRPS and RFE2 referenced against GPCC rainfall for the three wettest months at each pixel (2001–2010). (**a**,**b**) Correlation, (**c**,**d**); bias ratio, (i.e., the ratio between the mean of the validated product and mean GPCC precipitation); and (**e**,**f**) the mean absolute error (mm). Regions with average annual rainfall<50 mm are masked.

**Figure 3:** Correlation of near surface soil moisture (1992–2015, *n*=23) between CCI-SMv2.2 and Noah3.3+CHIRPS+MERRA-2 (0–10 cm). For the (**a**) East Africa, (**b**) Southern Africa, and (**c**) Western Africa domains. Regions with no vegetation are masked in the FLDAS estimates, and regions with dense vegetation are masked in the CCI-SMv2.2.

**Figure 4:** Correlation (r) of Percent of Normal (PON) Evapotranspiration (2003–2014, *n*=11) between the operational Simplified Surface Energy Balance (SSEBop) and Noah3.3+CHIRPS+MERRA-2. For the (**a**) East Africa, (**b**) Southern Africa, and (**c**) Western Africa domains.

**Figure 5:** February 2016 Percent of Normal ET from (a) Noah3.3+CHIRPS+MERRA-2 and (b) SSEBop.

**Figure 6:** Agricultural conditions for February 2016 represented by (a) End-of-Season Water Requirement Satisfaction Index (WRSI) anomalies and (b) drought classification based on February soil moisture percentile values. WRSI is the seasonal ratio of actual to reference evapotranspiration, and was computed with CHIRPS rainfall and USGS EROS reference ET derived from GDAS parameters. (**b**) Drought classification based on February soil moisture percentile values computed from Noah33+CHIRPS+MERRA-2 soil moisture (0–10 cm). The baseline period is 2000–2015. Severe drought is <20th percentile, drought is 20–30th percentile, abnormally dry is 30–45th percentile, normal is >the 45th percentile.

**Figure 7:** The Standardized Runoff Index (SRI) as an indicator of (a) short-term hydrological drought using 1-month (April 2016) aggregation, and (b) long-term hydrological drought using 24-month aggregation. Much of Southern Africa has been experiencing below average moisture conditions for at least 2 years, which is impacting reservoir water supplies.

**Figure 8:** VIC4.1.2 and Noah3.3 runoff with different meteorological inputs (CHIRPS+MERRA-2 and RFE2+GDAS). (**a**) SRI-24 averaged upstream Lake Kariba, on the border of Zambia and Zimbabwe. (**b**) SRI-24 averaged over Maputo Basin. The SRI-24 computed from Noah3.3 and VIC4.1.2 CHIRPS+MERRA-2 runoff show that 2015 is at or near record low levels experienced in 2004–05 and 1994–95. The RFE2+GDAS forced runs also shows low runoff in 2015 despite its relatively short record (2001-present) with respect to the 24-month integration period.

**Figure 9:** Screen-capture from the NASA Giovanni web tool used to extract and visualize data served on GES DISC. Note the selections of ‘Time Series: Seasonal’, December 1982–2015, ‘Keyword: FLDAS’, and selection of bounding box for spatial averaging.

**Figure 10:** Through NASA Giovanni, tabular data are easily and publicly accessible over the internet. Exports in MS Excel format can be used, for example, to (1) compute the z-scores of temperature and precipitation; (2) combine them into a drought index (rainfall—temperature; and (3) plot in rank order to visualize drought conditions during December of years from 1982–2015. For the domain selected, 2015 had the combined hottest and driest conditions on record. 2007 had the combined coolest and wettest conditions.

**Table 1:** FLDAS Specifications.

**Projection**	**Geographical latitude/longitude**
Land Surface Models	Noah3.3, VIC4.1.2
Spatial Extent	Centered on Continental Africa (40S, 20W; 40N, 55E)West Africa (5.3500 N, 18.65 W; 17.650 N, 25.850 E)East Africa (11.750S, 22.050E; 22.950N, 51.350 E)Southern Africa (37.850S, 6.050 E; 6.350N, 54.550 E)
Spatial Resolution	0.1 degree (Noah3.3), 0.25 degree (VIC4.1.2)
Time Period	1982—present (CHIRPS+MERRA-2); 2001-present (RFE2+GDAS)
Temporal Resolution	30 min Noah3.3 model timestep; 1 h VIC4.1.2 model timestep; daily output fields
Forcing	Multiple datasets derived from satellite measurements and atmospheric analyses
Forcing Heights	2 m for air temperature and specific humidity, 10 m for wind
Elevation Definition	SRTM
Vegetation Definition	University of Maryland (AVHRR), 1 km (VIC4.1.2) NCEP-modified IGBP(MODIS), 1 km (Noah3.3)
Soils Definition	Hybrid STATSGO/FAO Soil Texture
Output Format	NetCDF

**Table 2:** Land surface Datasets.

**Dataset Type**	**Domain**	**Spatial resolution**	**Temporal resolution**	**URL**
University of Maryland Vegetation Classification	Global	1 km	Static	http://glcf.umd.edu/data/landcover/
NCEP IGBP Vegetation Classification (MODIS)	Global	1 km	Static	ftp://ftp.emc.ncep.noaa.gov/mmb/gcp/ldas/noahlsm/README
NCEP monthly albedo	Global	0.144 deg	Monthly	ftp://ftp.emc.ncep.noaa.gov/mmb/gcp/sfcflds/test/fixed/README_albedo_gfrac.txt;
NCEP monthly green fraction	Global	0.144 deg	Monthly	ftp://ftp.emc.ncep.noaa.gov/mmb/gcp/sfcflds/test/fixed/README_albedo_gfrac.txt; http://www.emc.ncep.noaa.gov/mmb/gcp/sfcimg/gfrac/index.html
Boston University Leaf Area Index (AVHRR)	Global	1 km	Monthly	http://cybele.bu.edu/modismisr/products/avhrr/avhrrlaifpar.html
Elevation Database from SRTM	Global	30 s	Static	http://www2.jpl.nasa.gov/srtm/
FAO Harmonized World Soil Database	Global	30 s	Static	http://webarchive.iiasa.ac.at/Research/LUC/External-World-soil-database/HTML/index.html

**Table 3:** Meteorological Inputs.

**Dataset name**	**Dataset type & parameter**	**Domain**	**Spatial resolution**	**Time record**	**Temporal resolution**	**URL**
NCEP's Global Data Assimilation System (GDAS)	Model DerivedMeteorology Forcing	Global	Gaussian, time varying. Currently lat/long ~0.205°	Jan 2000—Current	3-hourly	http://www.emc.ncep.noaa.gov/index.php?branch=GFS
NASA's Modern Era Reanalysis (MERRA2)	Model DerivedMeteorology Forcing	Global	0.5° latitude×0.625° longitude	Jan 1980—current	hourly	https://gmao.gsfc.nasa.gov/reanalysis/MERRA-2/
NOAA CPC Africa Rainfall Estimation Algorithm v2 (RFE2)	Merged Satellite/ GaugeMean rain rate	20W-55E, 40S-40N	lat/lon, 0.1°	Jan 2001—Current	daily	http://www.cpc.noaa.gov/products/international/data.shtml
Climate Hazards Group InfraRed Precipitation with Station data (CHIRPS)	Merged Satellite/ GaugeMean rain rate	180W—180E, 50S-50N	lat/lon, 0.05°	Jan 1981—Current	daily	http://chg.geog.ucsb.edu/data/chirps/

**Table 4:** Routine FLDAS outputs and units available from the NASA GES DISC.

**Models**	**Model output description**	**units**
Noah3.3 & VIC4.1.2	Near surface wind speed	m s^−1^
Noah3.3 & VIC4.1.2	Near surface air temperature	K
Noah3.3 & VIC4.1.2	Net short wave radiation flux	W m^−2^
Noah3.3 & VIC4.1.2	Surface downward shortwave radiation	W m^−2^
Noah3.3 & VIC4.1.2	Total precipitation rate	kg m^−2^ s^−1^
Noah3.3 & VIC4.1.2	Surface radiative temperature	K
Noah3.3 & VIC4.1.2	Baseflow-groundwater runoff	kg m^−2^ s^−1^
Noah3.3 & VIC4.1.2	Storm surface runoff	kg m^−2^ s^−1^
Noah3.3 & VIC4.1.2	Latent heat net flux	W m^−2^
Noah3.3 & VIC4.1.2	Sensible heat net flux	W m^−2^
Noah3.3 & VIC4.1.2	Heat flux	W m^−2^
Noah3.3 & VIC4.1.2	Specific humidity	Kg kg^−1^
Noah3.3 & VIC4.1.2	Surface pressure	Pa
Noah3.3 & VIC4.1.2	Net long-wave radiation flux	W m^−2^
Noah3.3 & VIC4.1.2	Downward long-wave radiation flux	W m^−2^
Noah3.3 & VIC4.1.2	Evapotranspiration	kg m^−2^ s^−1^
Noah3.3 & VIC4.1.2	Soil moisture percentile (0–10 cm)	%
Noah3.3 & VIC4.1.2	Soil temperature (0–10 cm)	K
Noah3.3	Soil temperature (10–40 cm)	K
Noah3.3	Soil temperature (40–100 cm)	K
Noah3.3	Soil temperature (100–200 cm)	K
Noah3.3 & VIC4.1.2	Soil moisture (0–10 cm)	m^3^ m^−3^
Noah3.3	Soil moisture (10–40 cm)	m^3^ m^−3^
Noah3.3	Soil moisture (40–100 cm)	m^3^ m^−3^
Noah3.3	Soil moisture (100–200 cm)	m^3^ m^−3^
VIC4.1.2	Soil temperature (10–160 cm)	K
VIC4.1.2	Soil temperature (160–190 cm)	K
VIC4.1.2	Soil moisture (10–160 cm)	m^3^ m^−3^
VIC4.1.2	Soil moisture (160–190 cm)	m^3^ m^−3^
